# Mining actionable combined high utility incremental and associated sequential patterns

**DOI:** 10.1371/journal.pone.0283365

**Published:** 2023-03-29

**Authors:** Min Shi, Yongshun Gong, Tiantian Xu, Long Zhao

**Affiliations:** 1 Department of Computer Science and Technology, Qilu University of Technology (Shandong Academy of Sciences), Jinan, China; 2 School of Software, Shandong University, Jinan, China; 3 School of Information and Control Engineering, Qingdao University of Technology, Qingdao, China; Sejong University, KOREA, REPUBLIC OF

## Abstract

High utility sequential pattern (HUSP) mining aims to mine actionable patterns with high utilities, widely applied in real-world learning scenarios such as market basket analysis, scenic route planning and click-stream analysis. The existing HUSP mining algorithms mainly attempt to improve computation efficiency while maintaining the algorithm stability in the setting of large-scale data. Although these methods have made some progress, they ignore the relationship between additional items and underlying sequences, which directly leads to the generation of redundant sequential patterns sharing the same underlying sequence. Hence, the mined patterns’ actionability is limited, which significantly compromises the performance of patterns in real-world applications. To address this problem, we present a new method named Combined Utility-Association Sequential Pattern Mining (CUASPM) by incorporating item/sequence relations, which can effectively remove redundant patterns and extract high discriminative and strongly associated sequential pattern combinations with high utilities. Specifically, we introduce the concept of actionable combined mining into HUSP mining for the first time and develop a novel tree structure to select discriminative high utility sequential patterns (HUSPs) for downstream tasks. Furthermore, two efficient strategies (i.e., global and local strategies) are presented to facilitate mining HUSPs while guaranteeing utility growth and high levels of association. Last, two parameters are introduced to evaluate the interestingness of patterns to choose the most useful actionable combined HUSPs (ACHUSPs). Extensive experimental results demonstrate that the proposed CUASPM outperforms the baselines in terms of execution time, memory usage, mining high discriminative and strongly associated HUSPs.

## Introduction

High utility sequential pattern (HUSP) mining [1–5] is a critical technique in data mining, which has widely applications in real-world scenarios such as E-commerce recommendation, healthcare data analysis and bioinformatics. For example, e-commerce merchants can analyze a large number of customer purchase records to find useful high utility sequential patterns (HUSPs) both from customers and merchants so that customers are able to select good products and merchants can obtain more profits. Then, the e-commerce site can provide customers with personalized services based on their attributes and online purchase steps, while optimizing the layout of the e-commerce site. In this way, the service quality and economic efficiency of the website can be significantly improved. Compared with traditional sequential pattern mining (SPM) [6–8], the purpose of HUSP mining is to identify patterns associated with high profits (i.e., high utility) to help make decisions and gain more profit in the business.

In the era of big data, some works e.g., USpan [9], HuspExt [10], HUS-Span [11], SU-Chain [12] in HUSP mining are proposed to intently reduce the computational complexity of algorithms and improve decision efficiency, but they ignore pattern correlations and thus leads to a large number of redundant patterns generation. Consequently, mined sequential patterns are not actionable; meanwhile, the real valuable patterns are ignored and concealed in thousands of patterns sharing the same underlying sequences. As shown in Fig 1, the pattern <(fertilizer, flowerpot, sprinkling kettle), peony> mined by [3, 4] is simultaneously sold out with a low probability although the profit of selling peony is relatively high. Another pattern <(fertilizer, flowerpot, sprinkling kettle), hibiscus flower>is a common combination, but the profit is declining. Such mined patterns would influence the product profits due to weak associations between items and sequences. In practice, it is critical to consider the pattern associations in HUSP mining.

**Fig 1:** An example of HUSP sharing the same underlying sequences.

At present, the study of pattern association in HUSP mining is still open and unexplored. For business purposes, managers develop combined product strategies to find products that are more profitable than others. These combined products will not be very valuable or common, but the additional product can have a positive association with the underlying product, which can boost profitability. The most intuitive strategy is to invoke the off-the-shelf pattern correlation strategies in actionable combined high utility itemset (ACHUI) mining [13–15]. Concretely, few algorithms, such as CUARM [16], MUAP [17] and HUIPM [18], propose the criterion based on utility and frequency (i.e., support) to select combined products with a strong association for decision-making. However, these criteria are not directly employed to mine actionable combined HUSPs (ACHUSPs) for the following reasons.

First, the definitions of these criteria are not applicable to actionable combined HUSP (ACHUSP) mining. Second, HUSP mining takes the itemsets’ order into account and an item may occur in different itemsets of a sequence. Accordingly, an item may have multiple different utility values. In contrast, in HUI mining, an item only appears once in an itemset and has only one utility value. Furthermore, HUSP mining algorithms are not suitable for mining ACHUSPs because they do not take the sequences’ association into account. They assume that the frequency of all items is the same and then many spurious and valueless patterns are discovered with HUSP mining.

To address these issues, this work suggests a novel algorithm to mine discriminative ACHUSPs and introduces a new high utility-association rule to capture pattern associations for removing redundant candidates. The contributions of this paper are listed below.

- We present a novel Actionable Combined Utility-Association Rule (CUAR), based on which we can generate a pattern set with high utility and strong association. This is the first attempt, to the best of our knowledge, to choose high utility patterns without loss of representativeness (i.e., strong association).
- We proposed a new interestingness based on association and utility, called Associated-Utility Growth (AUG), to help remove redundant patterns and select discriminative ones. Moreover, two parameters are introduced to measure the effect of the additional item on the utility and support of the derivative sequence.
- We propose a global-local strategy to effectively select the actionable combined HUSPs. From a global perspective, we identify all the clusters of utility incremental sequential pattern based on specific underlying sequences; based on each cluster of sequential patterns, we estimate each utility incremental sequential pattern’s interestingness from a local perspective.
- Extensive experimental results on six datasets indicate the usefulness and efficiency of the proposed method.

The rest of this paper is organized as follows. The related work is described in Related Work. The basic concepts and definitions of utility-based sequential pattern mining are covered in Problem Statement. The CUASPM algorithm is described in depth in The Proposed Algorithm. The experiment results are presented in Experiments. Finally, Conclusion and Future Work describes the conclusion and future work.

## Related work

### High utility sequential pattern mining

Since it was initially developed in website logs sequence mining [19], HUSP mining has been a recent method for improving pattern actionability [15]. Then, extensive research [20] has been done on the HUSP mining problem. Ahmed et al. introduced two innovative techniques [21], UL (UtilityLevel) and US (UtilitySpan), to successfully find HUSPs from a sequential database. And the efficiency of the US approach is better than that of UL with fewer candidates generated. Since the definition of HUSP used in [21] was too specific, the authors in [9, 22] simplified the utility calculation of sequences and proposed a maximum utility measure that selected the maximum utility of a sequence as its utility. Additionally, they also proposed sequence-weighted utilization (SWU) property to minimize the amount of search space and memory usage. Then, an effective approach, USpan [9], was described by Yin et al. to choose the HUSPs with maximum utility and a tree structure to store the sequences’ utility. This approach used two pruning strategies to remove the meaningless sequences. Lan et al. proposed a projection-based PHUS [22] method and presented an upper-bound model and indexing strategy to select the relevant sequences rapidly and reduce the search time. To rationalize and simplify the *minutil* threshold setting, Yin et al. proposed the concept of top-k HUSPs instead of setting minimum utility value and presented TUS [23] method to select top-k HUSPs. At various phases of the mining process, our approach used three measures to continuously raise and update the thresholds.

To improve the efficiency of HUSP mining, Alkan et al. presented a pruning measure based on CRoM strategy and HuspExt approach [10] to efficiently extract HUSPs. Wang et al. [11] presented HUS-Span algorithm and two pruning strategies to select all HUSPs, and they also presented TKHUS-Span algorithm and three searching strategies, i.e. GDFS, BFS and the combination of BFS and GDFS to extract top-k HUSPs. Le et al. proposed a pruning measure to eliminate non-HUSP and two algorithms named AHUS and AHUS-P [24] to efficiently select all HUSPs. Lin et al. proposed SU-chain [12] structure to store more significant information to efficiently obtain HUSPs. To save some sequence information, such as utility, location, and time order, Gan et al. suggested the utility-array, a compact data structure. They also proposed the ProUM method based on a projection strategy to greatly improve the effectiveness of mining HUSPs. At the same time, PUO and PUK strategies were presented to filter the hopeless candidates and thus narrow the search space. Nevertheless, the authors also presented HUSP mining with UL-list (HUSP-ULL) [4] to efficiently accomplish the task of HUSP mining, and the utility-linked (UL)-list structure expedited the utility calculation of candidates, which contained both the UP (utility and position) information and header table. Meanwhile, they designed the pruning strategies named LAR and IIP to reduce candidates and irrelevant items, which can prevent the generation of more unpromising candidate sequences.

Some studies are available on the applications of HUSP mining. To choose web access sequences, Ahmed et al. proposed the UWAS-tree and IUWAS-tree [25] structures. This method can efficiently deal with the sequences’ forward and backward references simultaneously. Shie et al. first introduced the concept of utility into mobile data mining and put forward two tree-based approaches [26] to mine mobile sequences with high utility. The tree structure can store information on locations, items, paths and utilities. Zida et al. proposed a one-phase method HUSRM [27] and a compact utility-table structure to select sequential rules with high utility. Zihayat et al. presented HUSP-Miner [28] method to mine HUSPs by scanning the database only once, which combines the concept of stream mining with HUSP mining. In addition, the authors also suggested the HUSP-tree and ItemUtilLists structures to store the fundamental information for HUSP. Two pruning strategies, SFU and SWU, were introduced to shrink the HUSP-Tree in order to prevent the generation of unpromising candidates. Kim et al. [29] presented an efficient algorithm based on a sliding window approach to discover high utility patterns. This approach divided the stream data into fixed-sized multiple batch data and processed differently the importance of each batch data in a window according to the added time using the decaying factor. Meanwhile, an efficient algorithm [30] was proposed to mine high average-utility patterns based on a sliding window. It scanned the stream data once by using a list structure and utilized a novel pruning technique to reduce the search space. Besides, authors suggested an efficient approach [31] for mining high-utility patterns with negative unit profits.

Utility pattern mining has been widely used in real applications. A novel technique [32] considering the noises was suggested to overcome the limitation of traditional high utility pattern mining approaches. It utilized a utility tolerance factor to extract approximate high utility patterns from a noisy database. After the HUOMI algorithm [33] was proposed, which used an optimized data structure and an improved pruning technique to respond to the dynamic environment promptly.

Most of these algorithms focus on identifying HUSP and improving the efficiency of HUSP mining. Although these approaches have applied some real-world scenarios, they ignore both the relationship between sequential patterns and the effect of extensions on candidate sequences.

### Combined pattern mining

The concept of the combined association rule was initially discussed in [34], and it was then expanded upon there. Combined rule mining was a feasible way to merge different features from two databases into one pattern or patterns, and it was not necessary to merge two databases in this process. Further, Cao et al. [35] proposed high-impact combined pattern mining which can mine exceptional patterns such as high frequent or infrequent patterns. These patterns can not be recognized by traditional methods which can only extract high frequent patterns and can reveal important business impacts in solving business problems. This method was only applied in the frequency-based framework. In order to find both high profit and effective pattern combinations, Yeh et al. presented BU-UFM [36] approach based on a utility-frequent mining model. However, the definition of utility in this approach was different and was only used to select patterns. This approach did not combine patterns with their frequencies and utilities.

Accordingly, Shao et al. proposed the actionable combined utility-association rule structure which considered the relationships between items and presented CUARM [16] algorithm to find interesting utility-association rules(UAR). This algorithm first used UP-Growth [37] method with UP-Tree and minimum utility (*minutil*=0) to get all itemsets as underlying itemsets and then used two factors, i.e., contribution and weight to extract the set of UAR from these itemsets. Then they also proposed the concept of utility growth and MUAP [17] algorithm to mine actionable patterns with high utility increment and high reliance. This algorithm used global and local strategies to select actionable patterns from underlying patterns.

Although some methods have been proposed to find combined patterns, few works take the interestingness of ACHUSPs into consideration, which will be explored in our work.

## Problem statement

In this section, we redefine the Associated-Utility Growth (AUG) Pattern and introduce the relevant definitions for discovering ACHUSPs.

### Definitions

Let *I* = {*i*_1_, *i*_2_, …, *i*_*n*_} be a finite set containing *n* different items. A *q-item* is expressed as (*i*_*k*_, *q*_*k*_) that represents the item *i*_*k*_ with its purchase quantity (internal utility) *q*_*k*_. A *q-itemset* *X* = [(*i*_1_, *q*_1_)(*i*_2_, *q*_2_)…(*i*_*n*_, *q*_*n*_)] is a collection of *q-items*. A *q-sequence* *s* = <*X*_1_, *X*_2_, …, *X*_*m*_> denotes the sorted list of *q-itemsets* *X*_*k*_(1 ≤ *k* ≤ *m*). The *q-sequence* database S, which includes five *q-sequences* and six items from *a* to *f*, is shown in Table 1. The quantity of *q-items* and *q-itemsets* in a *q-sequence*, respectively, determines its length and size. The profit (external utility) of each item appearing in Table 1 is shown in Table 2.

**Table 1:** Q-sequence database S.

SID	Q-sequence
*S*_1_	<[(*b*, 3)(*d*, 2)][(*a*, 1)(*c*, 4)][(*f*, 4)]>
*S*_2_	<[(*a*, 2)][(*b*, 2)(*d*, 3)(*e*, 3)][(*c*, 1)(*d*, 4)]>
*S*_3_	<[(*a*, 2)(*d*, 4)][(*b*, 3)(*e*, 5)]>
*S*_4_	<[(*a*, 1)(*b*, 4)][(*a*, 2)(*c*, 3)(*d*, 5)][(*a*, 4)(*c*, 2)(*e*, 1)]>
*S*_5_	<[(*b*, 2)(*e*, 2)][(*a*, 4)(*c*, 3)(*f*, 6)][(*b*, 3)(*c*, 4)(*e*, 3)]>

**Table 2:** External utility table.

item	*a*	*b*	*c*	*d*	*e*	*f*
**profit($)**	4	3	4	2	5	2

**Definition 1.** *The frequency or support of a sequence* *t* *is the number of* *q-sequence* *containing* *t* *in the* *q-sequence* *database* S *and is denoted as* *sup*(*t*).

Based on Table 1, *sup*(< *c* >) is 4, *sup*(< (*cd*) >) is 2.

**Definition 2.** *The utility of a* *q-item* *i*_*k*_ *in a* *q-itemset* *X* *is defined as*:

$$\begin{array}{c} u\left(i_{k},X\right)=q\left(i_{k},X\right)\times p\left(i_{k}\right), \end{array}$$ (1)

*where* *q*(*i*_*k*_, *X*) *represents the internal utility of* *i*_*k*_ *in* *X* *and* *p*(*i*_*k*_) *is the external utility of* *i*_*k*_.

**Definition 3.** *The utility of a* *q-itemset* *X* *in a* *q-sequence* *s* *is defined as*:

$$\begin{array}{c} u\left(X,s\right)=\sum_{i_{k}\in X\wedge X\in s}u(i_{k},X). \end{array}$$ (2)

**Definition 4.** *The utility of a* *q-sequence* *s* *in* *q-sequence* *database* S *is defined as*:

$$\begin{array}{c} u\left(s\right)=\sum_{X\in s\wedge s\in S}u(X,s). \end{array}$$ (3)

**Definition 5.** *The utility of a* *q-sequence* *database* S *is defined as*:

$$\begin{array}{c} u\left(S\right)=\sum_{s\in S}u(s). \end{array}$$ (4)

**Definition 6.** *Given two* *q-itemsets* *X* *and* *X*′, if there exists the same item with the same profit in *X* for any item in *X*′, *X* contains *X*′, denoted as *X*′ ⊆ *X*.

**Definition 7.** *Given two* *q-sequences* *s* = < *X*_1_, *X*_2_, …, *X*_*m*_ > and $s^{{}^{\prime }}=<X_{1}^{{}^{\prime }},X_{2}^{{}^{\prime }},...,X_{n}^{{}^{\prime }}>$, if there exists integers 1 ≤ *j*_1_ ≤ *j*_2_ ≤ … ≤ *j*_*n*_ ≤ *m* such that $X_{k}^{{}^{\prime }}\subseteq X_{j_{k}}$(1 ≤ *k* ≤ *n*), then *s*′ contains *s*′ ⊆ *s*.

**Definition 8.** *Given a sequence* *t* = < *w*_1_, *w*_2_, …, *w*_*m*_ > *and a* *q-sequence* *s* = < *X*_1_, *X*_2_, …, *X*_*n*_ >, if *n* = *m* *and the items in* *X*_*k*_ *are the same as the items in* *w*_*k*_ *for* 1 ≤ *k* ≤ *n*, *which means* *t* *matches* *s*, *denoted as* *t* ∼ *s*.

**Definition 9.** *The utility of a sequence* *t* *in a* *q-sequence* *s* *is defined as*:

$$\begin{array}{c} u\left(t,s\right)=max\{u\left(s^{{}^{\prime }}\right)|t∼s^{{}^{\prime }}\wedge s^{{}^{\prime }}\subseteq s\}. \end{array}$$ (5)

*t*′*s* *utility in q-sequence database* S *is defined as*:

$$\begin{array}{c} u\left(t\right)=\sum_{s\in S}\left\{u\left(t,s\right)|t∼s^{{}^{\prime }}\wedge s^{{}^{\prime }}\subseteq s\right\}. \end{array}$$ (6)

**Definition 10.** *Sequence* *t* *in* S *is a HUSP if and only if*

$$\begin{array}{c} u(t)\geq minutil, \end{array}$$ (7)

*where the minutil is the minimum threshold specified by users*.

**Definition 11.** *The sequence* *X*_0_ *is known as an **Underlying Sequence (US)**, which is invariant throughout all equations*. Δ*X*_*i*_ *is known as an **Additional Item (AI)** and* *X*_*i*_ *is known as a **Derivative Sequence (DS)** or **Combined Sequential Pattern***.

$$\begin{array}{c} \left\{ \begin{array}{c} X_{0}+\Delta X_{1}\to X_{a},\\ X_{0}+\Delta X_{2}\to X_{b},\\ ...\\ X_{0}+\Delta X_{n}\to X_{n}, \end{array}\right. \end{array}$$ (8)

*where* Δ*X*_1_ ∩ Δ*X*_2_…∩ Δ*X*_n_ = ⌀ *and* *X*_*a*_ ≠ *X*_*b*_…≠*X*_*n*_.

With the same *US*, different *AIs* can be combined to find a cluster of *DSs*, and ACHUSPs will be select for decision-making. One of the *DSs* with the same *US* has the highest utility, while the other *DSs* has a utility. This type of combined HUSPs can provide much more valuable information and supports for managers. For example, a manager may sell some combination productions with high profit, while the same products with other different goods can result in a drop or a rise in profit. Obviously, such kinds of combined productions with high utility are better suited for business decisions.

### Mining combined sequential pattern with utility increment and strong association

A sequence is called *Incremental Sequence* since the number of items will grow. As shown in Fig 2, the utility of incremental sequence is changing dynamically and irregularly, meaning that the sequence’s utility may increase or decrease as its length increases. The measure of utility does not apply to extract actionable HUSPs, which can be supplemented with sequence frequency. Therefore, a new method called Associated-Utility Growth (AUG) Sequential Pattern Mining is introduced to detect Association-Maximum Incremental Sequences (AMIS) and Utility-Increasing Incremental Sequences (UIIS). Here, the maximum association does not mean the most frequent sequence, but refers to that those items in the sequence have a reasonable relationship. In the same way, utility increasing means that the utility of the derivative sequence derived from the underlying sequence by attaching an additional item is changing dynamically. Whereafter, when a cluster of derivative sequences is extracted using combinations of the same underlying sequence and various additional items, the measure of AUG is used to select ACHUSPs, which takes into account both the high association between the underlying sequence and the additional item as well as the high utility growth from the underlying sequence to the derivative sequence.

**Fig 2:** Incremental sequences with utility dynamics.

## The proposed algorithm

In this section, the CUASPM algorithm is presented to mine actionable combined sequential patterns which are both high utility increment and strong association by recursively projecting the utility-linked (UL)-list [4] based on the prefix sequences. The UL-List structure is utilized to save the sequence data and prevent repeated scans of the original database. The search space for mining HUSP is represented by the lexicographic sequence tree (LS-Tree). To save unnecessary computational costs, two pruning strategies are introduced to avoid the generation of hopeless candidates. In addition, we give a global and local approach to identify the utility growth sequential patterns and measure the interestingness of each derivative sequence. The details of these methods are represented below successively in the next subsection.

### Lexicographic sequence tree

To represent and arrange the search space for *q-sequences*, a lexicographic sequence tree (LS-Tree) like USpan [9] is utilized. The *I-Concatenation* or *S-Concatenation* approach is used to create all nodes in this tree (except for the null root node), and they are all arranged alphabetically.

**Definition 12.** *Given a sequence* *t* *and an item* *i*, *the* *I-Concatenation* *of* *t* *with* *i* *is appending* *i* *to the last itemset of* *t*, *which is denotes as* < *t*⊕*i* > _*I*-*Concatenation*_. *The* *S-Concatenation* *of* *t* *with* *i* *is adding* *i* *to a new itemset that is appended after the last itemset of* *t*, *which is denoted as* < *t*⊕*i* > _*S*-*Concatenation*_.

For example, given a sequence *t* = < (*bc*) > and an item *d*, < *t*⊕*d* >_*I-Concatenation*_ = < (*bcd*) > and < *t*⊕*d* >_*S-Concatenation*_ = < (*bc*)*d* >. By performing *I-Concatenation*, the size of <*t*⊕*d*> remains unchanged. Otherwise, the size of < *t*⊕*d* > increases by one.

As shown in Fig 3, any node in the LS-Tree strand for a potential candidate in the search space of ACHUSPs. To retrieve the entire collection of ACHUSPs, the tree is traversed by utilizing the depth-first-search method.

**Fig 3:** A lexicographic sequence tree.

The HUSP mining is to identify the entire set of all HUSPs that satisfy the *minutil* threshold efficiently. The way to obtain the combined sequential patterns is to extract HUSPs first implemented by using HUSP-ULL [4] with *minutil* and then identify the actionable combined sequential patterns from it, among the *minutil* specified by users. In essence, the baseline approach is a method to keep track of all sequential patterns and their utility, which can be referenced for details of the method in [4].

### The utility-linked list structure

The utility-linked (UL)-list structure similar to HUSP-ULL [4] is introduced to maintain the utility and position information of each *q-sequence*. The *q-sequences* containing candidate node are transformed into a UL-list structure and appended to the node’s projection database. Based on the projected database of this node, its utility and upper bound can be efficiently determined.

The UL-list structure includes **Header Table** and **UP (utility and position) Information**. The distinct items in the transformed *q-sequence* are kept in the Header Table together with the positions of their first occurrences. The UP information records the item’s information in the *q-sequence*, including an **item**, the **item’s utility**, the **item’s remaining utility**, and the **next position of this item**. Take *q-sequence* *S*_4_ for example to explain the content of UL-list structure in Table 3 and other *q-sequences* are treated in the same way.

**Table 3:** The Utility-Linked (UL)-list structure of *S*_4_.

**UP Information**	< [(*a*, $4, $71, 3)(*b*, $12, $59, −)][(*a*, $8, $51, 6) (*c*, $12, $39, 7) (*d*, $10, $29, −)][(*a*, $16, $13, −)(*c*, $8, $5, −)(*e*, $5, $0, −)] >
**Header Table**	(*a*, 1)(*b*, 2)(*c*, 4)(*d*, 5)(*e*, 8)

The UL-list structure also saves time by speeding up the process of finding candidate items. For a sequence *t* = < *ac* >, the corresponding *q-sequence* matches in *S*_4_ are <(*a*, 1)(*c*, 3)>, < (*a*, 1)(*c*, 2) > and <(*a*, 2)(*c*, 2) >. This instance shows that a sequence *t* may have more than one match since an item may appear several times in a *q-sequence* with varying quantities. Therefore, the positions of the matches need to be extracted and saved to find candidate items for generating a new sequence. The **concatenation point** is interpreted as the position of the last item with each match, and the *pivot* is the first concatenation point. Thus, the three concatenation points of *t* in *S*_4_ are 4, 7, 7 and the *pivot* is 4. According to the definition, for *I-Concatenation*, the candidate items are in the same itemset as the concatenation points and behind the concatenation points. In the above example, that is {*d*, *e*}. For *S-Concatenation*, the candidate items are in the itemsets appearing behind the *pivot* in each *q-sequence*. In the above example, that is {*a*, *c*, *e*}. Although the above sequence *t* has three *q-sequence* matches, the utility of *t* is the maximum utility value in that *q-sequences*.

The UL-list structure can quickly discover the candidate items to generate new sequences and calculate the utilities and upper bounds of sequences. To reduce space consumption, the original database is preserved as UL-lists only once. This algorithm only builds the projected UL-lists for each projection step, not the projected sub-database. The UL-lists of (*k* + 1)-*sequence* are built by scanning the UL-lists of *k*-*sequence*. In addition, this algorithm will consume less memory since the initial UL-lists are divided into smaller ones that are projected on the sub-sequences.

### Pruning strategies

#### Utility upper bound pruning

To narrow the search space and maintain the downward closure property, the upper bound of candidates is calculated using the sequence weighted utilization (SWU) [4], allowing for the early elimination of hopeless candidates.

**Definition 13.** (*Sequence weighted utilization*, *SWU*) *The* *SWU* *of a sequence* *t in* S *is defined as*:

$$\begin{array}{c} SWU\left(t\right)=\sum_{s\in S}\left\{u\left(s\right)|t∼s^{{}^{\prime }}\wedge s^{{}^{\prime }}\subseteq s\right\}. \end{array}$$ (9)

For example in Table 1, *SWU*(< *ac* >) = *u*(*S*_2_) + *u*(*S*_4_) + *u*(*S*_5_) = 47 + 75 + 96 = 218.

**Theorem 1** *Given a* *q-sequence database* S , *and two sequences* *t*_1_ *and* *t*_2_, *if* *t*_2_ *contains* *t*_1_, *then* *SWU*(*t*_2_) ≤ *SWU*(*t*_1_).

**Theorem 2** *Given a* *q-sequence* *database* S *and a sequence* *t*, *it can be gained that*:

$$\begin{array}{c} u(t)\leq SWU(t). \end{array}$$ (10)

Theorems 1 and 2 can be proven directly from [4, 11]. To enhance the effectiveness of the proposed algorithm, the tighter upper bound based on the PEU model [4] is introduced to expedite the search process. The following introduces details.

**Definition 14.** (*Prefix extension utility*, *PEU*) *The PEU of a sequence* *t* *in a* *q-sequence* *s* *is defined as*:

$$\begin{array}{c} \begin{array}{cc} PEU(t,s) & =max\{u\left(s^{{}^{\prime }}\right)+u\left(<s-s^{{}^{\prime }}{>}_{rest}\right)|t∼s^{{}^{\prime }}\wedge s^{{}^{\prime }}\subseteq s\}, \end{array} \end{array}$$ (11)

*where* *u*(< *s* − *s*′ >_*rest*_) *is the sum of the utilities of the items behind* *s*′ *in s. The* *PEU* *of the sequence* *t* *in* S *is then*

$$\begin{array}{c} PEU\left(t\right)=\sum_{s\in S}\left\{PEU\left(t,s\right)|t∼s^{{}^{\prime }}\wedge s^{{}^{\prime }}\subseteq s\right\}. \end{array}$$ (12)

**Theorem 3** *Given a sequence* *t* *and* *t*′, if *t* *is a prefix of* *t*′ (i.e., *t* ⊆ *t*′, then *u*(*t*)′ ≤ *PEU*(*t*′) ≤ *PEU*(*t*).

*proof*. Since *t* is a prefix of *t*′, *t*′ can be divided into the prefix *t* and the extension item *i* such that *t* + *i* = *t*′.

$$\begin{array}{c} \begin{array}{cc} u(t^{{}^{\prime }},s) & =max\{u\left(s^{{}^{\prime }}\right)|t^{{}^{\prime }}∼s^{{}^{\prime }}\wedge s^{{}^{\prime }}\subseteq s\}\\ & \leq max\{u\left(s^{{}^{\prime }}\right)+u\left(<s-s^{{}^{\prime }}{>}_{rest}\right)|t^{{}^{\prime }}∼s^{{}^{\prime }}\wedge s^{{}^{\prime }}\subseteq s\}\\ & =PEU(t^{{}^{\prime }},s)\\ & =max\{u\left(s_{t}\right)+u\left(s_{i}\right)+u\left(<s-s^{{}^{\prime }}{>}_{rest}\right)|\\ & t∼s_{t}\wedge i∼s_{i}\wedge s^{{}^{\prime }}=s_{t}+s_{i}\}\\ & \leq max\{u\left(s_{t}\right)+u\left(<s-s_{t}{>}_{rest}\right)|t∼s_{t}\wedge s_{t}\subseteq s\}\\ & \leq PEU(t,s). \end{array} \end{array}$$

Thus, $u\left(t^{{}^{\prime }}\right)=\sum_{t^{{}^{\prime }}∼s^{{}^{\prime }}\wedge s^{{}^{\prime }}\subseteq s\wedge s\in S}u(t^{{}^{\prime }},s)\leq \sum_{t^{{}^{\prime }}∼s^{{}^{\prime }}\wedge s^{{}^{\prime }}\subseteq s\wedge s\in S}PEU(t^{{}^{\prime }},s)=PEU\left(t^{{}^{\prime }}\right)\leq \sum_{t∼s^{{}^{\prime }}\wedge s^{{}^{\prime }}\subseteq s\wedge s\in S}PEU(t,s)=PEU\left(t\right)$.

According to Theorem 3, the upper bound on the utility of any offspring of *t* can be expressed as PEU(*t*). As a result, it is safe to prune each of *t*’s descendant nodes, and the mining outcome is unaffected when PEU(*t*) < *minutil*.

**Theorem 4** *Given sequences* *t*, *t*′ and an extension item *i*, *t* + *i* = *t*′, then

$$\begin{array}{c} u\left(t^{{}^{\prime }}\right)\leq \sum_{s\in S}\left\{PEU\left(t,s\right)|t^{{}^{\prime }}∼s^{{}^{\prime }}\wedge s^{{}^{\prime }}\subseteq s\right\}. \end{array}$$

*proof*. Based on Theorem 3, *PEU*(*t*′, *s*) ≤ *PEU*(*t, s*) and *u*(*t*′, *s*) ≤ *PEU*(*t*′, *s*). Thus, $u\left(t^{{}^{\prime }}\right)\leq PEU\left(t^{{}^{\prime }}\right)=\sum_{s\in S}\left\{PEU\left(t^{{}^{\prime }},s\right)|t^{{}^{\prime }}∼s^{{}^{\prime }}\wedge s^{{}^{\prime }}\subseteq s\right\}\leq \sum_{s\subseteq S}\left\{PEU\left(t,s\right)|t^{{}^{\prime }}∼s^{{}^{\prime }}\wedge s^{{}^{\prime }}\subseteq s\right\}$.

Based on Theorems 3 and 4, we introduce look-ahead removing (LAR) and irrelevant item pruning (IIP) [4] to cut down on the number of candidate sequences and eliminate unpromising candidate items early.

#### Mining global utility incremental sequential pattern based on LS-Tree

LS-Tree: According to the method used to determine a sequence’s utility, the utility of a node in a particular branch changes dynamically, which implies that the utility increment may drop. Since our algorithm is on the basics of association rule mining and utility growth, any branches whose utility falls will be first excluded from the proposed LS-Tree. The first node whose the increment of utility is positive is the target of the pruning process, which begins the search. After the aforementioned processing, the reorganized tree is known as the LS-Tree, and it is displayed in Fig 3.

Each node *N* in this tree is composed of *q-sequence* and its utility. All nodes will be generated by using *I-Concatenation* or *S-Concatenation* strategy. To extract all the complete sets of ACHUSPs, the depth-first-search approach is introduced in traversing the LS-Tree.

When traversing to a node, the support and utility of candidate items and sequences can be discovered by scanning the corresponding projected database. And they are applied to calculate the factors *W* and *C*, respectively. The following subsection will introduce these factors.

#### Mining locally interesting sequential pattern from clusters of DSs

According to global utility incremental sequences, those sequences are divided into clusters of actionable combined sequential patterns, which are composed of several derivative sequences including the same underlying sequences as well as several additional items. The related details are described as Eq 8.

Since the frequency-based and utility-based sequential pattern mining frameworks identify many uninteresting patterns, we provide a combined mining strategy to find attractive sequential patterns which consider both frequency and utility. To select the actionable combined high utility incremental and associated sequential patterns, two parameters are introduced to evaluate the utility increment and the association relationship, which measure the interestingness of combined sequential patterns. Furthermore, a coefficient is used to balance the importance of two parameters in a combined sequential pattern. Therefore, in a cluster of derivative sequences, the combined pattern with the highest coefficient is selected as an actionable combined high utility incremental and associated sequential pattern.

**Definition 15.** *The* *contribution* *C*(Δ*X* ∣ *X*_0_) *of Additional Item* (Δ*X*) *to make utility growth from the Underlying Sequence* (*X*_0_) *to the Derivative Sequence is denoted as*:

$$\begin{array}{c} C\left(\Delta X|X_{0}\right)=\frac{e^{R}-e^{-R}}{e^{R}+e^{-R}}, \end{array}$$ (13)

*among*,

$$\begin{array}{c} R=\frac{u(X)}{u(X_{0})}. \end{array}$$ (14)

As demonstrated in Fig 2, the utility of derivative sequence is neither monotonic nor anti-monotonic with its length increasing due to the additional item. Thus, the logistic function in Eq 13 measures the importance of an additional item in the utility perspective which makes the underlying sequence transform the derivative sequence. However, even though the contribution is intended to assess if Δ*X* contributes significantly to the promotion of the utility from *X*_0_ to *X*, the rate *R* is still used to measure the contribution. In addition, Eq 15 is introduced to measure the co-occurrence frequency of the underlying sequence and an additional item.

**Definition 16.** *The* *weight* *W*(Δ*X*∣*X*_0_) *of an additional item to measure the co-occurrence frequency of the underlying sequence and additional item is denoted as*:

$$\begin{array}{c} W\left(\Delta X|X_{0}\right)=\frac{sup(X)}{sup(X_{0}\cup \Delta X)}, \end{array}$$ (15)

*where* *sup*(*X*) *is the support of derivative sequence* *X*, *and* *sup*(*X*_0_ ∪ Δ*X*) *is the support of either underlying sequence* *X*_0_ *or additional item* Δ*X*:

$$\begin{array}{c} sup\left(X_{0}\cup \Delta X\right)=sup\left(X_{0}\right)+sup\left(\Delta X\right)-sup\left(X\right). \end{array}$$ (16)

**Definition 17.** *The combined coefficient* *AUG*(Δ*X* → *X*_0_) *to measure the interestingness that is the degree of the effectiveness of manufacturing the derivative sequence from the underlying sequence is denoted as*:

$$\begin{array}{c} AUG\left(\Delta X\to X_{0}\right)=I_{1}C+I_{2}W, \end{array}$$ (17)

*where* *I*_1_ + *I*_2_ = 1, *and the value of* *I*_1_ *is specified by users, and another is* *I*_2_ = 1 − *I*_1_. *I*_1_ *and* *I*_2_ *reflect the importance of parameters* *C* *and* *W*, *respectively*.

This formula is the sum of the value of *C*(Δ*X*∣*X*_0_) in Eq 13 and the value of *W*(Δ*X*∣*X*_0_) in Eq 15. Despite the utility from the underlying sequence to the derivative sequence increases, it is insignificance whether the underlying sequence and the additional item have a weak correlation, which represents customers may not buy these products together in most cases. Therefore, the sequence with the higher *AUG* will be selected through our approach, which suggests that those products represented by this sequence are more likely to get attention and be bought together.

### CUASPM algorithm

In this section, a novel algorithm called CUASPM is presented to obtain the entire set of the actionable combined utility-association sequential patterns. For each sequence *t*, all the extension sequences *t*′ are recognised and their *AUG* values also are evaluated using Eq 17. Only the most effective pattern will be chosen from the combined sequential patterns cluster which is formed in Eq 8.

**Algorithm 1 CUASPM**

**Input**: A quantitative sequential database S; a utility table *utable*; the minimum utility threshold, *minutil*.

**Output**: The set of *ACHUSPs*.

1: Scan S once to:1) calculate the *SWU*(*t*) and *u*(*t*) for each 1-*sequence* *t*; 2) calculate *u*(*s*) for each *s* ∈ *S*;

2: Get the revised database $S^{{}^{\prime }}$ by deleting the 1-*sequences* that *SWU*(*t*) < *minutil*;

3: Scan the revised database $S^{{}^{\prime }}$ once to construct the UL-List of each $s\in S^{{}^{\prime }}$;

4: **for** each 1-*sequence* *t* in $S^{{}^{\prime }}$ **do**

5:  *t.PD*←{the UL-list of $s|t\subseteq s\wedge s\in S^{{}^{\prime }}\}$;

6:  **Project-Mining**(*t*, *t.PD*, *ACHUSPs*);

7: **end for**

8: **return** *ACHUSPs*;

The pseudo-code of the **CUASPM** algorithm is described in the procedure of Algorithm 1. The SWU and utility values of each 1-*sequence* *t* and utility value of each sequence *s* are first gained by scanning the quantitative sequential database S (Line 1). The revised database $S^{{}^{\prime }}$ is then established by eliminating the 1-*sequences* that *SWU*(*t*)<*minutil* (Line 2). Then, the revised database $S^{{}^{\prime }}$ is once again scanned to create the UL-List of each $s\in S^{{}^{\prime }}$ (Line 3). For each 1-*sequence* *t* in $S^{{}^{\prime }}$, the algorithm creates the projected database *t.PD* to store its UL-lists containing utility and position information (Lines 4 to 5). After that, the **Project-Mining** procedure regards the candidate *ACHUSP* *t* as a prefix for mining other *ACHUSPs* with its projected database(Line 6). Last, the CUASPM algorithm returns the total ACHUSPs (line 8).

**Algorithm 2 Project-Mining(**(*t*, *t.PD*, *ACHUSPs*)

**Input**: prefix sequence *t*; projected database of *t*.

**Output**: The set of *ACHUSPs*.

1: *MAX_AUG*=0;

2: *ECMP*=None;

3: *t.PD*←IIP(*t.PD*); ← evaluated using IIP

4: Scan *t.PD* to find *C*^*I*^; ←evaluated using LAR

5: **for** each item *i* in *C*^*I*^ **do**

6:  *t*′ ← *I-Concatenation*(*t, i*);

7:  **Judge** (*t*′,*t.PD*, *MAX AUG*, *ECMP*, *ACHUSPs*);

8: **end for**

9: Scan *t.PD* to find *C*^*S*^;←evaluated using LAR

10: **for** each item *i* in *C*^*S*^ **do**

11:  *t*′ ← *S-Concatenation*(*t, i*);

12:  **Judge**(*t*′,*t.PD*, *MAX AUG*, *ECMP*, *ACHUSPs*);

13: **end for**

14: *ACHUSPs*←*ACHUSPs* ∪ *ECMP*;

The **Project-Mining** (Algorithm 2) procedure enumerates combined sequential patterns by utilizing the *I-Concatenation* and *S-Concatenation* operations. It first initializes two variables, *MAX AUG* = 0 and *ECMP* = None (Lines 1 to 2). The proposed IIP strategy is applied to evaluate whether the candidate items are relevant to generate new sequences. After eliminating irrelevant items, the UL-list is recalculated (Line 3). Then, the set of candidate items (i.e., *C*^*I*^ and *C*^*S*^) will be obtained from the reduced projection database *t. PD* by using LAR strategy, which is used for *I-Concatenation* and *S-Concatenation* (Lines 4 and 9). The *t.PD* is utilized to calculate the upper bounds of the candidate items generating a new sequence with prefix sequence. Based on the proposed LAR pruning strategy, the algorithm will discard the candidate item whose upper bound is below the *minutil* threshold. The new sequence is generated by performing *I-Concatenation* and *S-Concatenation* (Lines 6 and 11). Then, the **Judge** procedure is used to evaluate the new sequences (Lines 7 and 12), which will be further explained later. The algorithm ends when no candidates are generated. Last, ECMP is added to the set of ACHUSPs (Line 14).

**Algorithm 3 Judge**(*t*′,*t.PD*,*MAX AUG*, *ECMP*, *ACHUSPs*)

**Input**: prefix sequence *t*′; projected database of *t*; *MAX AUG*, *ECMP*, *ACHUSPs*.

1: Construct *t*′*.PD*←{the UL-list of *s* | *t*′ ⊆ *s* ∧ *s* ∈ *t.PD* };

2: Calculate *u*(*t*′), *PEU*(*t*′) and *sup*(*t*′);

3: **if** *PEU*(*t*′) ≤ *minutil* **then**

4:  **Project-Mining**(*t*′, *t*′*.PD*, *ACHUSPs*);

5:  **if** *u*(*t*′) ≤ *minutil* & *u*(*t*′) ≤ *u*(*t*) **then**

6:   Calculate the values of *t*′.*C* and *t*′*W*;

7:   Calculate the value of *t*′*.AUG*;

8:   **if** *t*′*.AUG* > *MAX_AUG* **then**

9:    *MAX_AUG*=*t*′*.AUG*;

10:    *ECMP*=*t*′;

11:   **end if**

12:  **end if**

13: **end if**

The **Judge** (Algorithm 3) procedure provides the main steps to measure the AUG values of candidate sequences. It first constructs the projected database *t*′*.PD* by scanning *t.PD* (Line 1). At the same time, the utility, *PEU*, and support of *t*′ are calculated to determine whether it is a *ACHUSP* (Line 2). If the *PEU* of *t*′ is no less than *minutil*, the **Project-Mining** procedure is applied to identify additional *ACHUSPs* by utilizing *t*′ and its projected database (Lines 3 to 4). If the utility of *t*′ is no less than the *minutil* threshold and larger than *t*, then the values containing *t*′.*C*, *t*′.*W*, and *t*′*.AUG* are calculated (Lines 5 to 7). If the value of *t*′*.AUG* is larger than *MAX AUG*, then the value of *MAX AUG* is equal to *t*′*.AUG* and the value of *ECMP* is *t*′ (Lines 8 to 11).

## Experiments

### Experimental settings

All the compared algorithms are implemented in Java. The experiments are conducted using a 64-bit Microsoft Windows 10 operating system and an Intel(R) Core(TM) i7–6700 @ 3.40 GHz with 40 GB of RAM.

The six datasets including real-life data and synthetic data are applied for the experiments, which are described in Table 4. The real datasets are *SIGN*, *FIFA*, *Yoochoose-buys* and *BMSWebView*2, and the synthetic datasets are *SynDataset*-40*K* and *SynDataset*-160*K*. These data can be found at https://www.philippe-fournier-viger.com/spmf/index.php?link=datasets.php and http://www.Almaden.ibm.com/cs/quest/syndata.html. Several experiments are conducted on these datasets to testify to the effectiveness and efficiency of the proposed CUASPM algorithm.

**Table 4:** Characteristics of the datasets.

Dataset	#Size	#Item	#Avg. seq length	#Avg. ele length	#Type
SIGN	730	267	52.0	1	Dense
FIFA	20, 450	2, 990	34.74	1	Dense
Yoochoose-buys	234, 300	16, 004	1.13	1.97	Sparse
BMSWebView2	77, 512	3, 340	4.62	1	Sparse
SynDataset-40K	40, 000	7, 537	6.20	4.32	Sparse
SynDataset-160K	159, 501	7, 609	6.19	4.32	Sparse

In general, the comparative evaluation indicators of the utility-based sequential mining algorithm include efficiency analysis with execution time and memory usage, effectiveness analysis with derived patterns. In the following subsections, these indicators are introduced to evaluate the performance of CUASPM. For efficiency analysis, ProUM [3] and the state-of-the-art HUSP-ULL [4] algorithms are selected as the baselines.

Next, the results of comparing derivative sequences (DSs) with the traditional HUSPs, frequent sequences (FSs) and underlying sequences (USs) respectively are presented. This part of the experiments are carried out as follows. Firstly, we collect the traditional HUSPs from each dataset together with their utilities and frequencies separately through HUSP-ULL. Secondly, we also collect all FSs with their frequencies and utilities using PrefixSpan [7]. Then we calculate both utilities and frequencies of the DSs, which are selected as ACHUSPs. At last, we draw the utilities and frequencies of the USs, DSs, HUSPs and FSs as shown in Figs 7 and 8. The purpose of comparing our algorithm with FS and HUSP mining is to demonstrate the ACHUSPs, which are both at high utility and high frequency.

### Datasets

In this subsection, we introduce four real-life datasets [38] and one synthetic dataset [39] to conduct experiments for evaluating the performance of the proposed algorithm. Table 4 gives detailed characteristics of these datasets.

- SIGN is a real dataset transformed from sign language utterance and contains approximately 730 sequences and 267 distinct items.
- FIFA is a click stream data that originates from number one the FIFA World Cup 98 website. It contains 20, 450 sequences and 2, 990 items and a dense data.
- Yoochoose-buys is a commercial dataset made up of a number of retail sessions, each of which contains the click events.
- BMSWebView2 is a click stream data from a webstore, which is used in KDD-Cup 200 [40] and is a collection of 77, 512 sequences containing 3, 340 different items.
- SynDataset is a kind of synthetic dataset generated by the IBM Quest Dataset Generator [39]. SynDataset-40K and SynDataset-160K are part of the synthetic dataset, which contain 40, 000 and 159, 501 sequences, respectively.

### Execution time

In this section, we conduct a series of experiments to compare the execution time of the CUASPM, the state-of-the-art algorithms, ProUM and HUSP-ULL. Fig 4 shows the execution time of those algorithms to verify the efficiency of CUASPM with *I*_1_ = 0.01. The experimental results demonstrate that CUASPM outperforms the contact algorithms for all datasets, which suggests that the pruning strategies can avoid generating more unpromising sequences and save time in finding ACHUSPs. For example, the ProUM algorithm takes more than 1, 000 seconds to discover all HUSPs in SynDataset-160K dataset, while CUASPM and HUSP-ULL only spend around 200 seconds in some cases. It is also observed that the CUASPM takes thousands of seconds to extract ACHUSPs in the FIFA dataset, whereas ProUM needs to take tens of thousands of seconds. Moreover, note that the CUASPM is closed to HUSP-ULL in terms of execution time. This is reasonable since CUASPM introduces the concept of actionable combined mining into HUSP-ULL to select fewer but more valuable ACHUSPs. Generally, the execution time of the algorithm decreases due to the *minutil* threshold increases. However, the execution time of CUASPM only changes slightly as the *minutil* threshold increases or decreases, which indicates that CUASPM is more stable than ProUM.

**Fig 4:** Execution time under the various *minutil* thresholds. (a) SIGN, (b) FIFA, (c) Yoochoose-buys, (d) BMSWebView2, (e) SynDataset-40K, and (f) SynDataset-160K.

### Memory usage

To show good efficiency and effectiveness, we compare the memory usage of three algorithms during their execution on real-life and synthetic data. Fig 5 gives the memory usage of CUASPM, HUSP-ULL and ProUM under the various *minutil* thresholds when *I*_1_ is 0.01. Overall, in some cases, there is little difference in memory usage between the three algorithms. For example, SIGN, SynDataset-40K and SynDataset-160K. For other datasets, the CUASPM algorithm consumes less memory than other algorithms since it generates fewer candidates.

**Fig 5:** Memory usage under the various *minutil* thresholds. (a) SIGN, (b) FIFA, (c) Yoochoose-buys, (d) BMSWebView2, (e) SynDataset-40K, and (f) SynDataset-160K.

### The number of pattern

Since CUASPM introduces the concept of actionable combined mining into HUSP-ULL to select ACHUSPs, we conduct experiments to discover the number of patterns for three algorithms with *I*_1_ = 0.01, and six datasets are used for comparisons by setting different *minutil* thresholds. As shown in Fig 6, we can obverse that the number of patterns extracted by CUASPM is always less than HUSP-ULL and ProUM for all datasets. The 1-*sequences* are abandoned in the process of discovering ACHUSPs since it is not significant to study the occurrences of 1-*sequences* in real life. Besides, for each candidate sequence, only one new sequence generated by the candidate sequence with different additional items will be selected, which caters to both high frequency and high utility. Thus, CUASPM can obtain patterns that are composed of utility growth and high association combinations.

**Fig 6:** The number of pattern under the various *minutil* thresholds. (a) SIGN, (b) FIFA, (c) Yoochoose-buys, (d) BMSWebView2, (e) SynDataset-40K, and (f) SynDataset-160K.

### Evaluation of the utility incremental

To demonstrate how utility increases from the underlying sequence (US) to the derivative sequence (DS), we select the top 100 ACHUSPs of each algorithm in each dataset for experiments, and those patterns are sorted in descending order by the utility of DSs. Table 5 indicates the parameter settings of the six datasets with *I*_1_ = 0.01. Fig 7 gives the utilities of the top 100 patterns (i.e., DSs) and their parent nodes (i.e., USs). The performance in SIGN, FIFA and synthetic datasets are much better than in Yoochoose-buys and BMSWebView2. The experimental results show that the selected pattern by performing CUASPM is a utility growth pattern from the underlying sequence to the derivative sequence. In conclusion, for each dataset, the increment of utility is positive, which means that the utility actually increases from the underlying sequence to the derivative sequence.

**Fig 7:** Utility incremental with *I*_1_ = 0.01. (a) SIGN, (b) FIFA, (c) Yoochoose-buys, (d) BMSWebView2, (e) SynDataset-40K, and (f) SynDataset-160K.

**Table 5:** The parameters setting.

Dataset	*minutil*
SIGN	0.012
FIFA	0.02
Yoochoose-buys	0.00024
BMSWebView2	0.0023
SnyDataset-40K	0.0006
SynDataset-160K	0.0006

### Evaluation of the frequency and utility

In this section, we have collected the frequencies and utilities of traditional HUSPs, FSs and ACHUSPs to illustrate the significance of the experiment in the form of a line chart. Here, the six datasets are used to obtain those patterns using HUSP-ULL, PrefixSpan and CUASPM with *I*_1_ = 0.01, and the corresponding parameter *minutil* setting is shown in Table 5.

First, HUSPs obtained by executing the HUSP-ULL algorithm are arranged in descending order of utilities, the top 100 patterns are selected and their support values are output. We compare the frequency of ACHUSPs and HUSPs to obverse the cooccurrence relationship between items. Second, all FSs are extracted by performing the PrefixSpan algorithm and sorted in descending order of supports. Then, the top 100 FSs with their utility are used to measure the sequence associations for high utility items, which are selected PrefixSpan algorithm.

By analyzing the frequency and utility, ACHUSPs are both high utility and strongly associated, which consider the correlation and utility increments between additional items and the underlying sequence. Fig 8 shows that most ACHUSPs have higher frequencies than HUSPs discovered by traditional HUSP mining. In the meantime, most ACHUSPs are much higher utility than FSs. For example, in SIGN and FIFA datasets, the CUASPM performs much better than that of HUSP-ULL and PrefixSpan. However, the performance of CUASPM is not so good in Yoochoose-buys and BMSWebView2. Generally, ACHUSPs can provide more valuable information and high probability for decision-making, which are both high utility and strongly associated.

**Fig 8:** Experiments for FSs, HUSPs and ACHUSPs with *I*_1_ = 0.01. (a) SIGN, (b) SIGN, (c) FIFA, (d) FIFA, (e) Yoochoosebuys, (f) Yoochoose-buys, (g) BMSWebView2, (h) BMSWebView2, (i) SynDataset-40K, (j) SynDataset-40K, (k) SynDataset-160K, and (l) SynDataset-160K.

### Evaluation of *I*_1_

Since the CUASPM algorithm requires a user-defined value of *I*_1_, we test the effect of different *I*_1_ values on four datasets, SIGN, FIFA, Yoochoose-buys and BMSWebView2. *I*_1_ and *I*_2_ are a pair of related parameters to measure utility growth and co-occurrence frequency, which reflect the importance of the contribution and weight of additional items, respectively. As shown in Fig 9, the experimental results can be observed that when *I*_1_ is set to 0.5 and 0.9 respectively, the utility of the former is less than or equal to the latter, while the comparative results of frequency are opposite, for example, SIGN and FIFA. But, the CUASPM in Yoochoose-buys and BMSWebView2 does not perform well. The frequency and utility of ACHUSPs found with different *I*_1_ are almost unchanged. Therefore, it can be found that the CUASPM algorithm is not sensitive to *I*_1_.

**Fig 9:** The influence of *I*_1_. (a) SIGN, (b) SIGN, (c) FIFA, (d) FIFA, (e) Yoochoose-buys, (f) Yoochoose-buys, (g) BMSWebView2, (h) BMSWebView2, (i) SynDataset-40K, (j) SynDataset-40K, (k) SynDataset-160K, and (l) SynDataset-160K.

## Conclusion and future work

In this paper, we provide a novel algorithm to mine a pattern set with high utility and strong association by considering item associations and the utility implied among the items. Specifically, we propose a new actionable combined Utility-Association approach to learn the associations between the items and sequence. Based on association and utility, we introduce new interestingness (i.e., AUG) to remove redundant patterns. Two parameters also are utilized to measure the utility increment and the association relationship. Furthermore, a global and local paradigm is proposed to optimize the selection process, which also prevents the generation of redundant candidate sequences. The experimental results demonstrate that our method can identify patterns with both incremental utility and high representativeness. More importantly, this is the first attempt to select high utility patterns without losing the representativeness, which is validated in the experiments.

We focus on the history of events in this work to mine HUSPs, and we leave the dynamics of events in HUSP in future work.

In the future, we will consider introducing the concept of actionable combined mining into high utility negative sequential pattern mining [31, 41–44] to discover combined negative sequential patterns, which can offer more useful information for decision-making.

## Supporting information

S1 Datasets Data sets are used in the experimental part to verify the effectiveness of the algorithm. (ZIP)
